RETRACTED

# Effects of Dietary Fiber Interventions on Glycemic Control and Weight Management in Diabetes: A Systematic Review of Randomized Controlled Trials

**DOI:** 10.7759/cureus.78497

**Published:** 2025-02-04

**Authors:** Syed Ali Hussein Abdi, Syed Imran Ali Abdi, Mohamed H Ali, Noor A Balani, Nazik A Balani, Hestia L Jacob, Ariana Seyfi, Gadeer H Al Shabout, Dena N Hamza, Alan Deiar Al-Talabani, Ramadan Khan

**Affiliations:** 1 Internal Medicine, Ajman University, Ajman, ARE; 2 Medicine, Gulf Medical University, Ajman, ARE; 3 Medicine, Thumbay University Hospital, Ajman, ARE; 4 Surgery, Ajman University, Ajman, ARE; 5 Medicine and Surgery, Ajman University, Ajman, ARE; 6 Internal Medicine, D.G Khan Medical College, Dera Ghazi Khan, PAK

**Keywords:** diabetes, dietary fiber, fasting plasma glucose, glycemic control, gut microbiota, hba1c, randomized controlled trials, resistant starch, systematic review, weight management

## Abstract

This systematic review explores the impact of dietary fiber interventions on glycemic control and weight management in individuals with diabetes or at risk for diabetes. A comprehensive search was conducted across PubMed, Embase, and Cochrane Library following the Preferred Reporting Items for Systematic reviews and Meta-Analyses (PRISMA) guidelines, identifying randomized controlled trials published in the last five years. Ten studies met the inclusion criteria, evaluating various types of dietary fiber, including soluble, insoluble, viscous fiber, and resistant starch. The findings demonstrated significant improvements in key glycemic markers such as fasting plasma glucose, glycated hemoglobin (HbA1c), and postprandial glucose levels, as well as weight management outcomes such as reductions in body weight and waist circumference. Secondary benefits included improvements in lipid profiles, insulin sensitivity, and gut microbiota composition. The quality assessment revealed a low risk of bias in most studies, ensuring robust evidence. Despite these promising results, gaps in long-term effects and variations in intervention efficacy warrant further research. These findings emphasize the potential of dietary fiber as a practical and accessible intervention in diabetes management and prevention.

## Introduction and background

Diabetes mellitus (DM) is a complex metabolic disorder characterized by chronic hyperglycemia resulting from defects in insulin secretion, insulin action, or both [1]. As the global prevalence of diabetes continues to rise, particularly type 2 DM (T2DM), there is an urgent need for effective interventions to manage the disease and prevent its complications [2]. Among the numerous factors influencing diabetes management, dietary interventions play a critical role. Specifically, dietary fiber, a type of carbohydrate that resists digestion and absorption in the small intestine, has gained increasing attention for its potential benefits in glycemic control and weight management, two crucial aspects of diabetes care [3]. The therapeutic effects of dietary fiber stem from its ability to modulate postprandial glucose levels, improve insulin sensitivity, and influence satiety, ultimately supporting glycemic stability and weight regulation [4].

RETRACTED

Numerous clinical trials have explored the impact of dietary fiber on metabolic outcomes, revealing a significant reduction in glycated hemoglobin (HbA1c), fasting blood glucose levels, and body weight among individuals with diabetes. The mechanisms underlying these benefits include delayed gastric emptying, reduced glucose absorption, and alterations in gut microbiota composition, which collectively contribute to improved metabolic health [5]. In addition, the incorporation of dietary fiber into a structured weight management program has shown promise in mitigating the risk of cardiovascular complications associated with diabetes. Despite these findings, the heterogeneity of fiber types, intervention strategies, and clinical outcomes across studies underscores the need for a systematic evaluation of evidence to draw definitive conclusions about the efficacy of fiber-based interventions in diabetes care.

To systematically evaluate the outcomes of dietary fiber interventions in glycemic control and weight management for individuals with diabetes, this review is guided by a clearly defined Population, Intervention, Comparator, Outcome (PICO) framework [6]. The population of interest includes adults with diabetes, encompassing type 1 diabetes, type 2 diabetes, and prediabetes, as defined by established diagnostic criteria. The intervention focuses on dietary fiber supplementation or dietary strategies that incorporate fiber, including specific types such as soluble fiber, insoluble fiber, or resistant starch. The comparator includes standard dietary advice, low-fiber diets, or placebo interventions. The primary outcomes assessed are changes in glycemic control markers, such as HbA1c, fasting blood glucose, and postprandial glucose, along with weight management outcomes, including body weight, BMI, and body fat distribution. This systematic review seeks to address the question: “What are the effects of dietary fiber interventions on glycemic control and weight management in individuals with diabetes compared to standard care or placebo interventions?” By synthesizing evidence from high-quality randomized controlled trials (RCTs), this review aims to provide valuable insights into the clinical efficacy of dietary fiber and its potential role in diabetes management guidelines.

RETRACTED

## Review

Materials and methods

Search Strategy

The search strategy for this systematic review was meticulously designed to ensure a comprehensive and unbiased collection of relevant studies. Following the Preferred Reporting Items for Systematic reviews and Meta-Analyses (PRISMA) guidelines [7], we conducted a structured search across multiple databases, including PubMed, Embase, and Cochrane Library. Keywords and MeSH terms related to dietary fiber, glycemic control, weight management, and diabetes were used, alongside Boolean operators to refine the search. Filters were applied to include only RCTs published in the last five years, in English, and involving human subjects. Duplicates were removed, and the remaining studies were screened based on predefined inclusion and exclusion criteria. Full-text articles were assessed for eligibility to ensure they addressed the research question. This rigorous and transparent search process aimed to minimize bias and enhance the reliability of the findings.

Eligibility Criteria

To ensure the inclusion of high-quality and relevant studies, this systematic review applied predefined eligibility criteria [8]. Only RCTs published in English within the last five years were considered, focusing on dietary fiber interventions in the context of glycemic control and weight management in individuals with diabetes or those at risk of developing the condition. Eligible populations included adults diagnosed with type 1 or type 2 diabetes, prediabetes, or gestational DM (GDM). Interventions were required to involve dietary fiber supplementation or fiber-enriched diets, including specific types such as soluble fiber, insoluble fiber, viscous fiber, or resistant starch. Comparators included placebo, standard care, or alternative dietary strategies without fiber emphasis.

The primary outcomes of interest were changes in glycemic markers, including fasting plasma glucose (FPG), HbA1c, and postprandial glucose levels, as well as weight management outcomes such as body weight, BMI, or body fat distribution. Secondary outcomes included lipid profiles, insulin sensitivity, and inflammatory markers. Studies were excluded if they were not RCTs, focused on pediatric populations, or combined dietary fiber with interventions that confounded the effects, such as pharmacological agents not consistent across study arms. This rigorous eligibility framework ensured the inclusion of robust, high-quality evidence directly addressing the research objectives.

Data Extraction

Data extraction for this systematic review was conducted using a standardized and pre-tested data extraction form to ensure consistency and accuracy. Key information collected from each study included author details, year of publication, study design, population characteristics, sample size, type and dosage of dietary fiber intervention, comparator details, outcome measures (e.g., glycemic control and weight management), and key findings. Extracted data also included study duration, adherence rates, and any reported adverse events. The process was performed independently by two reviewers, with discrepancies resolved through discussion or consultation with a third reviewer. This meticulous approach ensured that all relevant data were captured systematically, facilitating a comprehensive synthesis of the evidence and minimizing the risk of bias in data interpretation.

RETRACTED

Data Analysis and Synthesis

Data analysis and synthesis were conducted systematically to integrate findings from the included studies and address the research question. A qualitative synthesis was performed to summarize and compare outcomes such as glycemic markers (HbA1c, fasting glucose, and postprandial glucose), weight management parameters (body weight, BMI, and body fat distribution), and secondary outcomes like lipid profiles and inflammation. Heterogeneity among studies, including variations in population characteristics, intervention types, and study durations, was considered during synthesis. Subgroup analyses were explored where feasible, focusing on specific types of dietary fiber or distinct populations, such as those with type 2 diabetes versus prediabetes. A narrative approach was used to highlight trends, patterns, and differences in outcomes across studies, providing a nuanced understanding of the evidence base. This method ensured a robust and coherent summary of findings, offering valuable insights into the efficacy of dietary fiber interventions in diabetes management.

Results

Study Selection Process

The study selection process adhered to a rigorous and transparent methodology as outlined in Figure 1. An initial search across three major databases - PubMed, Embase, and Cochrane Library - yielded 497 records. After removing 88 duplicate entries, 409 unique records were screened based on their titles and abstracts. Of these, 132 records were excluded for not meeting the inclusion criteria. The remaining 277 full-text reports were sought for retrieval, but 158 could not be retrieved due to unavailability or access issues. Subsequently, 119 full-text reports were assessed for eligibility, resulting in the exclusion of 42 studies that were not RCTs, 33 studies that focused on pediatric populations, and 34 studies with combined interventions that confounded the effects of dietary fiber. Ultimately, 10 studies met all the inclusion criteria and were included in the final systematic review, as depicted in Figure 1. This rigorous process ensured the inclusion of high-quality evidence directly addressing the research objectives.

RETRACTED

**Figure 1:** PRISMA flow diagram illustrating the study selection process PRISMA: Preferred Reporting Items for Systematic reviews and Meta-Analyses

Characteristics of the Selected Studies

The characteristics of the selected studies, as summarized in Table 1, demonstrate a diverse range of populations, interventions, and outcomes that collectively provide robust insights into the role of dietary fiber in glycemic control and weight management. The studies predominantly included adults with type 2 diabetes, prediabetes, or related metabolic conditions, with sample sizes ranging from small pilot trials to larger RCTs. Interventions varied across studies, encompassing soluble and insoluble fiber supplementation, fiber-enriched diets, and co-administration with other bioactive compounds such as ginseng and probiotics. Comparators typically included placebo, standard dietary advice, or low-fiber diets. The outcomes assessed included key glycemic markers such as FPG, HbA1c, and postprandial glucose, as well as secondary outcomes like body weight, lipid profiles, and gut microbiota composition. Collectively, these studies highlight the potential of dietary fiber to improve metabolic health across diverse clinical settings while revealing variations in effectiveness depending on fiber type, population characteristics, and study design.

**Table 1:** Summary of the study designs, population demographics, dietary fiber interventions, comparators, primary and secondary outcomes, and key findings from RCTs included in this systematic review 2h PG: 2-hour plasma glucose; CONGA: continuous overall net glycemic action; cT2-DDAS: contextual type 2 diabetes distress assessment system; DMS: digestible maize starch; FMT: fecal microbiota transplantation; FPG: fasting plasma glucose; GCT: glucose challenge test; GDM: gestational diabetes mellitus; GRADE: glycemic risk assessment diabetes equation; HbA1c: hemoglobin a1c (glycated hemoglobin); HDL: high-density lipoprotein; HMS: high-amylose maize starch; IGT: impaired glucose tolerance; LDL: low-density lipoprotein; NAFLD: non-alcoholic fatty liver disease; NBS: native banana starch; PGX®: PolyGlycopleX (a proprietary soluble fiber supplement); RCT: randomized controlled trial; RS: resistant starch; T2D: type 2 diabetes; T2DM: type 2 diabetes mellitus

Author(s) and year	Study design	Population	Intervention	Comparator	Outcome(s)	Key findings
Basu et al. (2021) [9]	RCT	Women with obesity at high risk of GDM (n = 34; mean age: 27 ± 5 years; BMI: 35.5 ± 4.0 kg/m²)	280 g of whole blueberries and 12 g of soluble fiber daily for 18 weeks	Standard prenatal care with nutrition education	Gestational weight gain, glycemic control (blood glucose via GCT), and inflammation (CRP levels)	The intervention group showed lower gestational weight gain (6.8 ± 3.2 kg vs. 12.0 ± 4.1 kg, P = 0.001), reduced blood glucose (100 ± 33 mg/dL vs. 131 ± 40 mg/dL, P < 0.05), and lower CRP levels (P = 0.002). No significant differences in lipid profiles or infant birth weight.
Li et al. (2024) [10]	RCT	Middle-aged and elderly prediabetic patients (n = 54; 27 in each group)	Daily dietary fiber supplementation (15 g mixed fiber per serving) for six months, followed by health education	Health education alone	Waist circumference, waist-to-hip ratio, FPG, 2h PG postprandial insulin, HbA1c, triglyceride/HDL ratio, and diabetes incidence	The intervention group showed significant reductions in FPG, 2h PG, postprandial insulin, and central obesity after six months compared to baseline. Lower HbA1c, triglyceride/HDL ratio, and diabetes incidence were observed compared to the control group. Benefits persisted at the 12-month follow-up.
Su et al. (2022) [11]	Controlled open-label trial	Adults with T2D	Specially designed diet combined with FMT for 90 days	Specially designed diet alone	Blood glucose, blood pressure, gut microbiota composition, BMI, and blood lipid profile	Both interventions improved glycemic control and blood pressure. FMT led to faster changes in gut microbiota composition, increasing beneficial bacteria like *Bifidobacterium* and reducing sulfate-reducing bacteria like *Bilophila *and *Desulfovibrio*. Improvements in blood glucose, BMI, and lipid profile were correlated with microbiota changes.
Liu et al. (2024) [12]	RCT (secondary analysis of the MARCH Trial)	Newly diagnosed Chinese T2DM patients (n = 551; 286 in the acarbose group and 265 in the metformin group)	Dietary fiber intake from various sources (whole grain, legume) over 48 weeks combined with acarbose or metformin monotherapy	Low-fiber diets or high-carbohydrate-low-fiber diets	Glycemic control, β-cell function, insulin sensitivity, weight loss, and HDL-C levels	Higher whole grain and total fiber intake improved β-cell function, insulin sensitivity, and glycemic control with acarbose. Legume fiber improved glycemic control in both groups but was associated with better weight loss only under metformin. High-carbohydrate-low-fiber diets worsened glycemic control under acarbose but improved insulin sensitivity and weight loss under metformin.
Frias et al. (2023) [13]	Double-blind RCT	Adults with T2D (n = 192; mean age: 54.3 years; mean HbA1c: 7.8%; mean BMI: 35.9 kg/m²)	Prebiotic fiber-enriched nutritional formula for 12 weeks	Placebo formula (fiber-absent) and non-blinded dietary advice-only group	Diabetes Distress Assessment System (cT2-DDAS), HbA1c, and gut microbiota composition	The intervention group showed significant reductions in cT2-DDAS (-0.4, p = 0.03) and HbA1c (-0.64%, p = 0.01) compared to placebo. An increased abundance of butyrate-producing bacteria (*Roseburia faecis* and *Anaerostipes hadrus*) was observed in the intervention group.
Arias-Córdova et al. (2021) [14]	Randomized crossover trial	Adults with T2D (n = 17; aged 28-65 years; BMI ≥ 25 kg/m²)	RS intake from NBS or HMS for four days	DMS	Glycemic control (fasting glycemia and 24-hour mean blood glucose) and glycemic variability (CONGA, GRADE, and J-index)	NBS reduced fasting glycemia changes compared to DMS (p = 0.0074). However, RS from HMS and NBS did not improve overall glycemic control or variability. Further studies are required to explore the impact of baseline microbiota and environmental factors.
Zurbau et al. (2021) [15]	Double-blind RCT	Adults with T2D (n = 104; mean age: 59 years; mean BMI: 29.0 kg/m²; mean HbA1c: 7.0%)	Co-administration of 10 g viscous fiber, 60 g white chia seeds, and ginseng extracts (1.5 g American and 0.75 g Korean red) for 24 weeks	Energy- and fiber-matched control (53 g oat bran, 25 g inulin, 25 g maltodextrose, and 2.25 g wheat bran)	HbA1c, body weight, and dietary adherence	The intervention group had a significant reduction in HbA1c compared to the control (-0.27%, p = 0.03). Greater reductions were observed in participants with baseline HbA1c > 7% (-0.56%, p = 0.07). Body weight and diet remained unchanged. Interventions were well tolerated with no adverse events.
Reimer et al. (2021) [16]	Double-blind RCT	Adults with overweight/obesity and T2D (n = 290; baseline HbA1c: 7.2 ± 1.1% in the intervention group and 7.0 ± 0.9% in the placebo group)	Soluble viscous fiber supplement (PGX®, 15-20 g/day) as an adjunct to a medically supervised weight management program for 52 weeks	Isocaloric placebo (rice flour, 6.4-8.6 g/day) with a weight management program	HbA1c, weight loss, waist circumference, LDL cholesterol, and gut microbiota composition	PGX group showed a significant reduction in HbA1c (-0.23%) at 52 weeks compared to baseline, with no between-group difference. Significant reductions in body weight and waist circumference occurred only in the PGX group. PGX also reduced LDL cholesterol and increased the abundance of beneficial gut microbiota (*Collinsella*, *Parabacteroides*, and *Roseburia*).
Kabisch et al. (2021) [17]	RCT	Adults with IGT (n = 180; subgroup for MRI analysis: n = 47)	Insoluble cereal fiber supplementation for two years	Placebo supplementation	Body fat distribution (visceral and hepatic fat), fasting glucose, HbA1c, insulin resistance, and inflammation	Fiber supplementation reduced visceral and non-visceral fat, fasting glucose, HbA1c, fasting insulin, and uric acid in the fiber group. No significant between-group differences were observed after adjusting for weight loss. A trend for liver fat reduction in individuals with NAFLD was noted in the fiber group.
Mitchell et al. (2015) [18]	RCT	Adults at risk for T2D (n = 48; aged 40-75 years)	Prebiotic supplementation with inulin (10 g/day) for six weeks	Placebo supplementation	Insulin sensitivity, skeletal muscle metabolic flexibility, intestinal permeability, serum endotoxin levels, inflammation, endothelial function, arterial stiffness, and fecal bacterial composition	Hypothesized that inulin supplementation improves insulin sensitivity and metabolic flexibility and reduces inflammation. Study design emphasized controlled feeding to minimize dietary confounding. Results have yet to confirm efficacy, but they aim to inform clinical dietary recommendations for reducing cardiometabolic risk in prediabetes.

Quality Assessment

The quality assessment of the included studies, as detailed in Table 2, reflects a generally robust methodological standard, with the majority of studies demonstrating a low risk of bias across key domains. Randomization processes were well-conducted in all studies, ensuring balanced allocation of participants to intervention and control groups. Most studies showed a low risk of deviations from intended interventions, with adherence to protocols and minimal contamination between groups. Measurement of outcomes was also consistently robust, with clear definitions and reliable tools used across studies. However, some concerns were noted in domains such as missing outcome data and selection of reported results, particularly in studies with smaller sample sizes or open-label designs, such as Su et al. [11] and Arias-Córdova et al. [14]. Despite these minor limitations, high-quality trials like those by Basu et al. [9], Frias et al. [13], and Reimer et al. [16] provided strong evidence with complete data reporting and minimal risk of bias, enhancing the reliability of the review’s conclusions.

RETRACTED

**Table 2:** Evaluation of methodological quality and risk of bias for the included studies, based on randomization processes, adherence to interventions, outcome measurement, and reporting consistency RCT: randomized controlled trial

Study	Randomization process	Deviations from intended interventions	Missing outcome data	Measurement of outcomes	Selection of reported results	Overall risk of bias	Comments
Basu et al. (2021) [9]	Low risk	Low risk	Low risk	Low risk	Low risk	Low risk	Well-conducted RCT with appropriate randomization and complete data reporting
Li et al. (2024) [10]	Low risk	Low risk	Some concerns	Low risk	Low risk	Some concerns	Some missing follow-up data in the control group, but unlikely to affect results
Su et al. (2022) [11]	Some concerns	Low risk	Some concerns	Low risk	Low risk	Some concerns	Open-label design introduces potential bias; missing data from microbiota analysis
Liu et al. (2024) [12]	Low risk	Low risk	Low risk	Low risk	Some concerns	Low risk	Results robust, but secondary analysis limits control over initial design decisions
Frias et al. (2023) [13]	Low risk	Low risk	Low risk	Low risk	Low risk	Low risk	Double-blind design with high adherence and complete outcome reporting
Arias-Córdova et al. (2021) [14]	Low risk	Low risk	Some concerns	Low risk	Low risk	Some concerns	Small sample size and short duration may affect generalizability
Zurbau et al. (2021) [15]	Low risk	Low risk	Low risk	Low risk	Low risk	Low risk	High-quality trial with detailed reporting and no major concerns
Reimer et al. (2021) [16]	Low risk	Low risk	Low risk	Low risk	Low risk	Low risk	Large sample size and robust design; long duration adds reliability
Kabisch et al. (2021) [17]	Low risk	Low risk	Some concerns	Low risk	Low risk	Some concerns	Long duration, but effects confounded by weight loss adjustments
Mitchell et al. (2015) [18]	Low risk	Low risk	Some concerns	Low risk	Low risk	Some concerns	Small sample size; controlled feeding minimizes confounding but limits generalizability

Discussion

The systematic review revealed consistent evidence supporting the positive effects of dietary fiber interventions on glycemic control and metabolic health in various populations, including those with type 2 diabetes, prediabetes, and GDM. Across studies, dietary fiber supplementation, either as standalone interventions or adjuncts to pharmacological or dietary regimens, demonstrated significant reductions in key glycemic markers such as FPG, HbA1c, and postprandial glucose levels. For instance, Basu et al. [9] showed that soluble fiber and blueberry supplementation significantly reduced blood glucose levels and inflammation in pregnant women at high risk of gestational diabetes, while Li et al. [10] reported sustained improvements in HbA1c and diabetes incidence among prediabetic patients after six months of daily mixed-fiber supplementation.

Several studies highlighted the interplay between dietary fiber and gut microbiota in enhancing glycemic control. For example, Su et al. [11] and Frias et al. [13] demonstrated that fiber-enriched nutritional formulas and diets combined with fecal microbiota transplantation led to favorable shifts in gut microbial composition, correlating with improvements in metabolic outcomes such as HbA1c and BMI. Additionally, studies examining specific fiber types, such as resistant starch [14] and viscous fiber [15,16], highlighted their distinct mechanisms in improving glycemic and lipid profiles. Notably, while most studies showed significant benefits of fiber supplementation, some, like Kabisch et al. [17], observed limited effects on visceral and hepatic fat after adjusting for weight loss, indicating that the magnitude of benefits may vary based on individual metabolic characteristics and baseline conditions. These findings underscore dietary fiber’s critical role in improving glycemic control and its potential as a cornerstone in managing and preventing diabetes.

RETRACTED

The findings of this systematic review align with the existing literature, which consistently highlights the benefits of dietary fiber in glycemic control and metabolic health [19]. Previous systematic reviews and meta-analyses have documented reductions in HbA1c, fasting glucose, and postprandial glucose levels with fiber supplementation, supporting its role as a non-pharmacological strategy for managing diabetes [20]. However, some nuances emerged in this review. For example, while most studies confirmed significant improvements in glycemic markers, others, like Kabisch et al. [17], observed limited effects on visceral and hepatic fat, suggesting that fiber’s metabolic benefits might be influenced by baseline weight loss or fat distribution. Furthermore, the observed synergy between fiber supplementation and gut microbiota modulation, as reported by Su et al. [11] and Frias et al. [13], adds a novel dimension to the current understanding, indicating a microbiome-mediated mechanism. Variations in outcomes across studies may be attributed to differences in population characteristics (e.g., age, BMI, and glycemic status), fiber types (e.g., soluble vs. insoluble, resistant starch), and intervention durations. These differences underscore the importance of tailored fiber interventions to maximize therapeutic benefits across diverse patient populations [21].

The findings of this systematic review underscore the potential of dietary fiber as a practical and accessible intervention for improving glycemic control and metabolic health, particularly in individuals with diabetes or at risk for the condition [22]. Incorporating dietary fiber into routine dietary recommendations could serve as a complementary strategy alongside pharmacological treatments, as it not only improves key glycemic markers like HbA1c and FPG but also offers additional benefits such as weight management and modulation of gut microbiota. For clinicians, the evidence supports recommending specific types of fiber, such as soluble fiber, viscous fiber, or resistant starch, tailored to the patient’s needs and preferences. On a broader scale, these findings could inform public health policies by advocating for increased fiber intake through dietary guidelines, nutrition education programs, and the development of fiber-enriched food products. Practical implementation in real-world settings, such as integrating fiber-focused counseling into diabetes management protocols, can empower patients to adopt sustainable dietary habits, potentially reducing the burden of diabetes-related complications.

RETRACTED

The observed benefits of dietary fiber in glycemic control and metabolic health can be attributed to several well-established biological and physiological mechanisms. Dietary fiber, particularly soluble and viscous types, slows gastric emptying and reduces postprandial glucose absorption by forming a gel-like matrix in the gut, thereby mitigating blood glucose spikes. Additionally, fiber fermentation in the colon produces short-chain fatty acids, such as butyrate, which improve insulin sensitivity and modulate inflammatory pathways [23]. The modulation of gut microbiota by fiber, highlighted in studies such as Su et al. [11] and Frias et al. [13], further supports its role in metabolic health by increasing beneficial bacterial populations like *Bifidobacterium *and *Roseburia*, while reducing harmful species linked to metabolic dysfunction. This microbiota shift enhances intestinal barrier function, reduces systemic inflammation, and positively influences lipid metabolism. Collectively, these mechanisms provide a theoretical framework explaining how fiber not only improves glycemic control but also contributes to broader metabolic and anti-inflammatory benefits, reinforcing its role in managing and preventing diabetes [24].

This systematic review has several strengths, including a rigorous search strategy that utilized multiple databases, comprehensive inclusion criteria focused on high-quality RCTs, and strict adherence to the PRISMA guidelines to ensure transparency and reproducibility. These methodological strengths enhance the reliability and validity of the findings. However, certain limitations must be acknowledged. The review may be subject to publication bias, as only studies published in English were included, potentially excluding relevant research in other languages. Additionally, heterogeneity in study populations, fiber types, and intervention durations posed challenges in synthesizing outcomes. Many included studies had small sample sizes or short follow-up periods, limiting the generalizability of the results and the ability to assess long-term effects. Despite these limitations, the findings provide valuable insights into the role of dietary fiber in glycemic control and metabolic health, highlighting the need for further large-scale, long-term trials.

RETRACTED

Despite the promising findings, several gaps in the evidence base warrant further investigation. Many studies included in this review were limited by short follow-up durations, making it difficult to assess the long-term effects of dietary fiber on glycemic control and metabolic outcomes. Future research should prioritize large-scale, long-term RCTs that explore the sustained impact of specific types of dietary fiber, such as resistant starch or viscous fiber, on diverse populations, including those with varying stages of glucose intolerance and different demographic or cultural backgrounds. Additionally, the role of fiber in modulating gut microbiota and its precise mechanistic pathways remain incompletely understood, requiring more advanced microbiome analyses and metabolomic studies. Investigating the synergistic effects of fiber with other dietary or pharmacological interventions could also provide a more comprehensive understanding of its therapeutic potential. Addressing these gaps will enhance the clinical applicability and generalizability of dietary fiber as a key intervention for diabetes management.

## Conclusions

This systematic review highlights the significant role of dietary fiber interventions in improving glycemic control and metabolic outcomes in individuals with diabetes and those at risk. The evidence demonstrates that dietary fiber, through mechanisms such as delayed glucose absorption, enhanced insulin sensitivity, and gut microbiota modulation, can effectively reduce key markers like HbA1c, fasting glucose, and postprandial glucose levels. These findings reinforce the importance of incorporating dietary fiber into routine dietary recommendations as a complementary strategy to pharmacological and lifestyle interventions. By addressing both short-term glycemic control and long-term metabolic health, dietary fiber offers a practical and impactful approach to managing and potentially preventing diabetes. Future research will further refine our understanding, but these findings already provide a robust foundation for integrating dietary fiber into diabetes care guidelines.
